The article "The utility of Jerk-locked back averaging technique in diagnosis of generalized myoclonic epilepsy with normal scalp EEG: A case report" was published in 2019. Journal: Medicine (Baltimore).

# The utility of Jerk-locked back averaging technique in diagnosis of generalized myoclonic epilepsy with normal scalp EEG: A case report

**DOI:** 10.1097/MD.0000000000014185

**Published:** 2019-01-18

**Authors:** Xiangyu Zheng, Zan Wang, Chang Liu, Minghui Hu, Yudan Lv

**Affiliations:** Department of Neurology, Department of Neurology and Neuroscience Center, The First Hospital of Jilin University, 71, Xinmin Street, Changchun, P. R. China.

**Keywords:** cortical origin, generalized seizure, Jerk-locked back averaging technique, myoclonus, scalp EEG

## Abstract

**Rationale:**

The diagnosis of myoclonic epilepsy and the classification of generalized or partial type may be challenging, especially when the scalp electroencephalogram (EEG) is normal. In such situation, how to apply another electrophysiological technique to begin the diagnosis and classification? The utility of Jerk-locked back averaging technique has been described in our case.

**Patient concerns:**

A Chinese patient (male, 21 years old) presented with frequent unilateral or bilateral shoulder-jerking. He has an epilepsy history of complex partial seizure (CPS) or secondary tonic-clonic seizure (sGTCS) for 10 years.

**Diagnosis:**

After admission, scalp EEG was performed with the normal result when the patient showed the jerks. According to the patient's clinical presentation, we suspected myolconic seizure, but there was lack of objective evidence. Then we used Jerk-locked back averaging technique to help begin the diagnosis. A bilateral-symmetrical time-locked, evoked cortical averaging potential that preceded the jerk has been found. So the jerks were considered as cortical origin and generalized myoclonic seizure was confirmed.

**Interventions:**

So in this situation, we added another antiepileptic drug of Levetiracetam (1500 mg/24 h).

**Outcomes:**

One week later, the jerk seizure had disappeared, and in the following visit, he had an improved prognosis with decreased seizure frequency.

**Lessons:**

Generalized polyspike-slow wave in EEG was common to see in myoclonic seizure and can help to make the classification. However, it should not dissuade clinicians from the diagnosis of myoclonic epilepsy with normal scalp EEG. Under this condition, we may apply other electrophysiological technique such as Jerk-locked back averaging technique, to give objective evidence to verify the cortical origin.

## 1 Introduction

Myoclonus is characterized by sudden, brief, shock-like involuntary movement, which presents as short jerk (10–100 ms) or rhythmic jerks.^[1]^ Myoclonus can occur at rest, during voluntary movement, or after stimuli. Myoclonus can be divided into cortical or subcortical jerk, and if the myoclonus is observed at rest, it usually has a strong association with some neurological diseases, such as epileptic disorders, spinal myoclonus, posthypoxic myoclonus, or Creutzfeldt–Jakob disease.^[2]^ Besides this, cortical myoclonus is the common subtype, if it is presented with generalized discharges in electroencephalogram (EEG), which implies myoclonic epilepsy.^[3]^

The technique of Jerk-locked back-averaging employs electromyography (EMG) electrodes for the arms or legs, and correlates averaged responses with EMG bursts used as a trigger. If a time-locked, evoked cortical averaging potential that precedes the EMG trigger was found, it means that the jerk was associated with cortical origin.^[4]^ So, Jerk-locked back-averaging technique has been shown to be useful not only for detecting EEG changes preceding myoclonus but also for investigating the relationship between the EEG and myoclonus that are not recognizable by routine EEG.

So far, the EEG has been considered as a valuable neurophysiological method in the evaluation and classification of myoclonic seizure. However, in some condition, jerks do not show a time-locked EEG discharge, so we may apply the Jerk-locked back-averaging technique to begin diagnosis. Additionally, whether such application can classify the seizure type as myoclonic epilepsy (generalized or partial) should be explored, which will have a direct effect on the treatment plan. In our case, we presented a patient with frequent unilateral or bilateral shoulder-jerking, and we applied the Jerk-locked back-averaging technique to establish the diagnosis of myoclonic epilepsy and make the classification. The patient has provided written informed consent and this case report has been approved by Research Ethics Board of the First Hospital of Jilin University.

## 2 Case presentation

A 21-year-old Chinese male patient has a history of epilepsy for 10 years. He presented with complex partial seizure (CPS) and secondary tonic-clonic seizure (sGTCS) with a frequency of 3–4 times a week. CPS was described as transient consciousness-lost companied with oropharynx automatism. He insisted on antiepileptic therapy of Oxcarbazepine (1200 mg/day) without improvement. In the past, he has given up the therapy of topiramate and valproic acid due to unsatisfactory effect. After this admission, his mother planned to make a schedule for epilepsy surgery. However, within 2 weeks recently, the patient developed another new seizure type of unilateral or bilateral-shoulder jerks frequently. In admission, physical examination was negative, then scalp EEG was performed, but with normal result. No synchronized, Jerk-locked spike or spike-slow wave has been found (Fig. 1). Magnetic resonance imaging (MRI) showed focal schizencephaly in right temporal-parietal lobe (Fig. 2). Mini-Mental State Examination (MMSE) score was 30/30. According to the patient's clinical seizure, we made a suspected diagnosis of myoclonic seizure but lacking objective evidence, and his MRI changes, previous seizure types should be considered carefully. In this situation, we need to explore another electrophysiological technique to help begin diagnosis. And we chose the Jerk-locked back-averaging technique, which employed EEG electrodes and EMG electrodes for the upper limbs (according to the 10/20 EEG system) and correlated averaged EEG responses with EMG bursts used as a trigger. In other words, we named the bilateral-shoulder jerks as EMG trigger point, made 15 times averaged superposition of Jerk-locked EEG before the trigger point. In order to ensure the data reliable, we applied 64-channel Event-related evoked potential machine produced by Neuroscan Compumedics Limited with a sampling rate of 1000 Hz. The filter setting was from 0.3 Hz to 70 Hz. The patient was tested in an electrically shielded room. During the data-processing, baseline correction, artifact rejection, filter settings, segmentation, and simple averaging were performed, respectively. After the examination, a time-locked, evoked negative cortical averaging potential that precedes the EMG activity has been found (Fig. 3), and was shown as symmetrical bilaterally in both hemisphere (Fig. 4), which was different from scalp-EEG (Fig. 1). The evoked EEG-potential began at 50 ms prior to the movement onset with amplitude of 6.5 and 7.5 μV. Such results may indicate: (1) bilateral-shoulder jerks were cortical myoclonus and may be myoclonic seizure probably; (2) such myoclonic seizure may be generalized. In order to verify such assumption, we named the unilateral-shoulder jerks as EMG trigger point, made the same analysis again, obtained the same result fortunately. Combining the suspected seizure with electrophysiological results described above, we made a clinical diagnosis of myoclonic epilepsy (generalized seizure). After the additional therapy of Levetiracetam (1.0 g/day) for 4 days, such bilateral-shoulder jerks have disappeared and sGTCS seizures have also decreased gradually. After the communication with the patient's family, they decided to give up the epilepsy surgery and insisted on antiepileptic drug. In the following visit, the patient had a better prognosis with low seizure frequency.

**Figure 1:** No synchronized, Jerk-locked spike or spike-slow wave has been found in scalp EEG.

**Figure 2:** Focal schizencephaly in right temporal-parietal lobe.

**Figure 3:** A time-locked, evoked negative cortical averaging potential precedes the EMG trigger.

**Figure 4:** Averaging potential is symmetrical bilaterally. Frontocentral averaging potentials have been marked as blue, green, purple, which have larger amplititudes. Bilateral averaging potentials in both sides are synchronized and symmetrical.

## 3 Discussion

As described in our case, the patient developed a special manifestation of unilateral or bilateral-shoulder jerks, but the scalp EEG was normal without synchronized discharges. How to make the diagnosis, epilepsy seizure, pseudoseizure, or dystonia? And the diagnosis will be closely related to the therapy and prognosis. Under this condition, other objective electrophysiological technique seems much more important. Commonly, EEG has been considered as a helpful tool in the diagnosis of myoclonic seizure, and polyspike-slow wave consisting of polyspikes followed by slow wave is usually characterized. However, in special cases, although the patient was presented with cortical myoclonic seizures, no synchronized discharges have been found in EEG. Such situation has also been described in previous study, and different jerks-amplitudes may be associated with different EEG discharges, such as no time-locked EEG discharges before or after the small-amplitude jerks, while generalized spike-wave bursts synchronized to the large-amplitude jerks.^[5,6]^ In our case, we obtained the similar results as that of the unilateral or bilateral-shoulder jerks seemed gently, and the amplitude shown in EMG was about 5–7 μV. When the jerking was presented without abnormal discharge in scalp EEG (Fig. 1), the myoclonic seizure should also be considered by clinicians.

According to the pathophysiologic mechanism, myoclonus is classified into three main categories: cortical, subcortical, and spinal. Cortical myoclonus shows a negative EEG shift preceding the jerks by a short interval. Subcortical-reticular myoclonus tend to be generalized including neck flexion, shoulder elevation, and knee extension, but with no time-locked discharges before the EMG event. Besides this, many patients with dystonia have brief muscle jerks repetitively, which can be distinguished from myoclonus due to the distinctive dystonic postures and absence in EEG shift preceding the jerks. Cortical myoclonus was very common to see in myoclonic seizure; such myoclonus can involve the whole body or partial limbs, and present as generalized or focal jerk. But both seizures are associated with abnormal discharges in EEG. So when the EEG was absent, the diagnosis and classification of myoclonic seizures may be challenging.

Under such condition, EEG-EMG Jerk-locked back-average technique may be useful for diagnosis and differential diagnosis. Bereitschafts potential (BP) is originally described as cortical potential preceding voluntary movements. The early BP is the initial slow rising segment and indicates the movement-preparation of the supplementary motor and premotor areas. The late BP is the steep rising segment, which starts about 400 ms prior to the movement onset and indicates the movement-selection and execution of contralateral motor cortex and premotor cortex.^[7,8]^ In prior studies, patients with motor tics had no BP prior to the movement, 86% of patients with functional myoclonus had early BP prior to the movement, cortical myoclonus had late BP with a short interval preceding the jerks,^[9,10]^ which can help to make differential diagnosis between functional myoclonus, motor tics, and cortical myoclonus. Besides this, we tried to explore the Jerk-locked back-average technique in the differential diagnosis of generalized or partial seizure type by comparing the symmetry of the lateral evoked-potentials from anterior lobe to posterior lobe.

However, there is an absolute limitation when applying the Jerk-locked back averaging to the patients with myoclonus as it is necessary to collect a sufficient number of jerks for making average analysis. When the jerks are too infrequent or too small to be picked up by the surface EMG, or when jerks occur too frequent (less than two seconds apart), this technique is not adequate.^[11]^ Therefore, this method is not always applicable to patients widely. Besides this, it is important to use the earliest muscle and not the later muscle for back-averaging so that we can see what is happening before movement.^[8]^ So there are selective indications for Jerk-locked back-average technique.

In conclusion, although the Jerk-locked back-average assessment of myoclonus is not as widely used as traditional EEG, however, under special situation, it may be an optional choice, and can give some contributions to clinician to make a proper diagnosis and optimal management.

## Acknowledgment

We thank Dr. Jiang Wu who was involved in the conceiving of manuscript or revising it critically for important intellectual content.

## Author contributions

XY Z has been involved in drafting the manuscript or revising it critically for important intellectual content; YD L have made substantial contributions to conception and design, or acquisition of data, or analysis and interpretation of data. All the authors have given the final approval of the version to be published. Each author has participated sufficiently in the work to take public responsibility for appropriate portions of the content and agreed to be accountable for all aspects of the work in ensuring that questions related to the accuracy or integrity of any part of the work are appropriately investigated and resolved.

**Conceptualization:** Yudan Lv, Xiangyu Zheng.

**Data curation:** Zan Wang.

**Formal analysis:** Chang Liu.

**Software:** Minghui Hu.

**Supervision:** Yudan Lv.

**Writing – original draft:** Yudan Lv.
